# Recommendation System for Privacy-Preserving Education Technologies

**DOI:** 10.1155/2022/3502992

**Published:** 2022-04-16

**Authors:** Shasha Xu, Xiufang Yin

**Affiliations:** Zhengzhou Preschool Education College, Zhengzhou, Henan 450000, China

## Abstract

Considering the priority for personalized and fully customized learning systems, the innovative computational intelligent systems for personalized educational technologies are the timeliest research area. Since the machine learning models reflect the data over which they were trained, data that have privacy and other sensitivities associated with the education abilities of learners, which can be vulnerable. This work proposes a recommendation system for privacy-preserving education technologies that uses machine learning and differential privacy to overcome this issue. Specifically, each student is automatically classified on their skills in a category using a directed acyclic graph method. In the next step, the model uses differential privacy which is the technology that enables a facility for the purpose of obtaining useful information from databases containing individuals' personal information without divulging sensitive identification about each individual. In addition, an intelligent recommendation mechanism based on collaborative filtering offers personalized real-time data for the users' privacy.

## 1. Introduction

Artificial intelligence-based educational techniques have advanced significantly in recent years, and their applications in various academic fields have increased. Implementing artificial intelligence in education encompasses a broad range of intelligent instructional and evaluation methods, including intelligent tutoring systems, intelligent performance assessment, intelligent virtual agents, talking robots, humanized chatbots, and any other approach based on artificial intelligence [1]. These classroom innovations can benefit a diverse range of students, particularly those with disabilities. Thanks to new intelligence technologies, these students now have a more flexible and personalized educational solution.

In general, artificial intelligence can be combined with other methods (e.g., speech recognition, machine vision, and disability assistant) to develop advanced tutor systems that can help students learn more effectively [2]. Furthermore, approaches based on artificial intelligence can be used to create adaptive and personalized learning systems that are tailored to the unique characteristics of each individual student.

Nevertheless, as AI models reflect the data over which they were trained, data that may have privacy or other sensitivities associated with it, they are vulnerable. This work proposes a privacy-preserving [3] recommendation system that uses differential privacy in this spirit. Differential privacy [4] is a technology that allows researchers and database analysts to acquire useful information from databases that contain people's personal information without disclosing the unique identify of the persons who have provided the information. Achieving this can be accomplished by including the bare minimum of distractions in the information provided by the database system. The amount of distraction introduced is significant enough to protect privacy while still allowing for the provision of information to analysts to continue to be valid. Differential privacy, in its most basic sense, is the process of forming data anonymously by deliberately adding noise into a dataset. Data analysts are capable of doing any and all possible (functional) statistical analysis without revealing any personal information.

Specifically, this study presents an innovative privacy-preserving recommendation system for educational technologies. It is a fully automated intelligent system that can categorize trainees based on their requirements and special skills. The abilities of each student are automatically categorized into one of several categories. Using a directed acyclic graph machine learning method, the model uses differential privacy in order to protect the private information of each individual learner. Also, an intelligent module based on collaborative filtering offers personalized real-time privacy recommendations.

Afterward, in Section 2, we learn about the proposed system's technique. Exemptions for applying the proposed method are outlined in Section 3.  Section 4 concludes by summarizing the findings and drafting the following potential directions for the work.

## 2. Proposed Methodology

A directed acyclic graph (DAG) [5] is used to express a probabilistic representation of the data structure created from the model and their putative independence. The classification method is then utilized to validate the whole combined probability distributions in the DAG [5]. The goal is to categorize an *X* sample into one of the supplied categories *C*_*1*_*, C*_*2*_*,…, C*_*n*_ using a probability model constructed according to Bayes theory in order to get the desired result. Overall, this is a first-level classification based on probabilities rather than predictions, a fact that has been demonstrated experimentally to be more useful, faster, and more efficient. In this case, projections are made to a certain extent, and the goal is to keep costs as low as possible. Each category is distinguished by a probability distribution that has occurred in the past. We assume that the sample *X* belongs to a class Ci, and we calculate the probability [5, 6] using the definitions and Bayes theory, respectively. To put it in another way, the initial step in the procedure is to understand how the pupils are dependent on one another and then assign probabilities to them, insuring how likely it is that their ability will change over time. As a result, the proposed system incorporates prior knowledge gathered from the model into the model learning process through a probabilistic representation of the data structure that arises for each learner, hence, enhancing the overall effectiveness of the system. A further consideration is the uncertainty in the model parameters that have been generated, which may be caused by noise such as a random or deceptive evaluation procedure, among other things.

In order to assess the overall performance, the following criteria of the DAG algorithm were used [7–9]:

(1) Overall accuracy (OvAc): this metric reflects the proportion of correctly identified samples in relation to the total number of test samples in a given period.
(2) Average accuracy (AvAc): this indicator displays the average accuracy of the different categories.
(3) Kappa rate: using the following function, we can determine how well the truth map and the final categorization map agree on various statistical criteria:
  (1) $$\begin{array}{c} K=\frac{p_{0}-p_{e}}{1-p_{e}}\\ =1-\frac{1-p_{0}}{1-p_{e}}, \end{array}$$
where *p*_*o*_ is the correlation between actual agreement and *p*_*e*_ is the theoretical likelihood of random agreement.
(4) McNemar test: to evaluate the significance of categorization accuracy derived from different methodologies, a McNemar test was used:
  (2) $$\begin{array}{c} z_{12}=\frac{f_{12}-f_{21}}{\sqrt{f_{12}+f_{21}}}, \end{array}$$
where *f*_*ij*_ samples accurately categorized in classification and *i* mistakenly classified in the other one *j*.
(5) Coefficient of determination, *R*^2^: use it to express correlation between two variables in percentage terms. The coefficient of determination is a measure of the degree to which the values of *X* and *Y* are correlated and calculated as follows:
  (3) $$\begin{array}{c} R^{2}=1-\frac{\sum_{i=1}^{n}{\left(Y_{i}-{\hat{Y}}_{i}\right)}^{2}}{\sum_{i=1}^{n}{\left(Y_{i}-{\underline{Y}}_{i}\right)}^{2}}, \end{array}$$
where *Y*_*i*_ are the actual values of the dependent variable, ${\hat{Y}}_{i}$ have been calculated based on our best estimates for this dependent variable, and *Y* is computed by taking the observed data and averaging it the number of observations.
(6) Root relative squared error (RRSE): in order for a model to be considered successful, the absolute correlation between predicted and actual values must be equal to zero:
  (4) $$\begin{array}{c} \text{RRSE}=\frac{\sum_{j=1}^{n}{\left(P_{\left(ij\right)}-T_{j}\right)}^{2}}{\sum_{j=1}^{n}{\left(T_{j}-\underline{T}\right)}^{2}}, \end{array}$$
where *P*_(*ij*)_ is the anticipated value for a simple hypothesis that the algorithm generates *j* and *T*_*j*_ and *T* are the desired value for the simple hypothesis *j*, with the following connection being used to determine:
  (5) $$\begin{array}{c} \underline{T}=\frac{1}{n}\sum_{j=1}^{n}T_{j}. \end{array}$$

In addition, the proposed method uses differential privacy. Before being shared through the suggested technique, personal data might be obscured by statistical noise that has been slanted in a certain direction. It is possible to see relevant information emerge when a huge number of people contribute the same information. Three ingredients—sensitive data, curators who need to provide statistics, and adversaries who want to retrieve the sensitive data—can all be solved through differential privacy. This reverse engineering is a type of privacy breach [3, 4, 10].

Finally, an intelligent recommendation memory-based approach was used to measure user privacy and compute the similarity between users [11, 12]. Finding persons with similar interests may be accomplished using the locality-sensitive hashing, which utilizes the closest neighbor algorithm in a linear time frame. A set of privacy restrictions is then proposed based on the *k* most comparable users and their related user-item matrices. Easy construction and usage, easy facilitation of new data, content-independent of the items being recommended, and effective scalability with co-rated goods are some of the advantages that this technique has to offer [13].

An abstract illustration of the proposed architecture is presented in Figure 1, which depicts as parts of a flowchart the basic steps of how the proposed system works.

## 3. Experiments

A preliminary exam for categorizing pupils' ability in their various level departments is the subject of this scenario. Students take this simple examination to determine their fitness to continue in higher-level education studies. It includes a set of questions or exercises evaluating skill or knowledge based on a scientific standard that can identify the real learning abilities of each learner [14–16]. Specifically, the preliminary test includes psychometric questionnaires and the purpose is to detect misunderstandings, ambiguities, disabilities, or other learning difficulties that may have the students.

The outcomes of this preliminary test are the dataset used by the classification algorithm. The dataset is used to contain ten questions that come from 350 volunteer students.  Table 1 presents the statistical analysis of the preliminary test used in this study.

The questionnaire is satisfactorily reliable in measuring the determination of students' moods and corresponding abilities and can be used for further processing by the proposed learning system [17, 18].

### 3.1. Step 1: Classification Process and Results

This model's probabilistic values and the abovementioned statistical analysis of the questions [19] map each student's reply to the DAG as a pair of variables based on these criteria [6] in form *B* = 〈G, Θ〉, where *G* is the nodes *Χ*_1_*, Χ*_2_*,…, X*_*n*_._._ In this form, each question in the questionnaire is represented as a probability value, along with its corresponding edge (the answers to each question). Graph *G* conveys the assumption that each variable *X*_*i*_ is independent of the inheritance assumed by *G*. Θ identifies the parameters of the network. Specifically, this set contains the parameter *θ*_*x*_*i*_*|π*_*i*__=*P*_*B*_(*x*_*i*_*|π*_*i*_) for each *x*_*i*_ implementation of *X*_*i*_ in the condition *π*_*i*_, for the set of *X*_*i*_ parents in G. Therefore, B defines a unique probability distribution over the variables, namely [5, 7, 20],

(6) $$\begin{array}{c} P_{B}=\left(X_{1},X_{2},\ldots ,X_{n}\right).=\prod_{i=1}^{n}P_{B}\left(\pi_{i}\right)\\ =\left.\prod_{i=1}^{n}\theta_{X_{i}}|\pi_{i}\right). \end{array}$$

There are three internally distinct paths linking two vertices *u* and *v* such that neither of them has the same orientation, or there are two directed cycles with a common vertex if there is a strong component, that is, neither a cycle or a single vertex. Number of predicted components is capped above [5, 20, 21]:

(7) $$\begin{array}{c} 2\left(\begin{array}{c} n\\ 2 \end{array}\right)\sum_{i=1}^{n}\sum_{j=1}^{n}\sum_{k=1}^{n}\left(\begin{array}{c} n\\ i \end{array}\right)i!p^{i+1}\left(\begin{array}{c} n\\ j \end{array}\right)j!p^{j+1}\left(\begin{array}{c} n\\ k \end{array}\right)k!p^{k+1}+\left(\begin{array}{c} n\\ 1 \end{array}\right)\sum_{i=2}^{n}\sum_{j=2}^{n}\left(\begin{array}{c} n\\ i \end{array}\right)i!p^{i+1}\left(\begin{array}{c} n\\ j \end{array}\right)j!p^{j+1}\leq \frac{\lambda^{3}}{n}\sum_{i=0}^{\infty }\sum_{j=0}^{\infty }\sum_{k=0}^{\infty }\lambda^{i+j+k}+\frac{\lambda^{2}}{n}\sum_{i=0}^{\infty }\sum_{j=0}^{\infty }\lambda^{i+j}=O\left(n^{-1}\right). \end{array}$$

Based on the Markov inequality, there are no such components. So, we can bound the expected number of cycles of length larger than *ω* by

(8) $$\begin{array}{c} \sum_{k=\omega }^{n}\left(\begin{array}{c} n\\ k \end{array}\right)\left(k-1\right)!p^{k}=\sum_{k=\omega }^{n}\frac{\prod_{i=0}^{k-1}\left(n-i\right)}{n^{k}}\frac{\lambda^{k}}{k}\leq \sum_{k=\omega }^{n}\lambda^{k}=O\left(\lambda^{\omega }\right). \end{array}$$

To compute the expectation of *X*_*n*_, we have

(9) $$\begin{array}{c} E\left[X_{n}\right]=\sum_{k=3}^{n}\left(\begin{array}{c} n\\ k \end{array}\right)\left(k-1\right)!p^{k}. \end{array}$$

It follows that

(10) $$\begin{array}{c} \underset{n⟶\infty }{\lim}E\left(X_{n}\right)=\underset{n⟶\infty }{\lim}\sum_{k=3}^{n}\frac{\prod_{i=0}^{k-1}\left(n-i\right)}{n^{k}}\frac{\lambda^{k}}{k}∼\sum_{k=3}^{\infty }\frac{\lambda^{k}}{k}\\ =-\log\left(1-\lambda \right)-\lambda -\frac{\lambda^{2}}{2}\\ =a\left(\lambda \right). \end{array}$$

The *r*th factorial moment of *X*_*n*_ is

(11) $$\begin{array}{c} E\left[{\left(X_{n}\right)}_{r}\right]=\hat{\theta }\sum_{k_{1}=3}^{n}\sum_{k_{2}=3}^{n-k_{1}}\ldots \sum_{k_{r}=3}^{n-\sum_{i=1}^{r-1}k_{i}}\left(\begin{array}{c} n\\ k_{1},k_{2},\ldots ,k_{r},n-k_{1}-\ldots -k_{r} \end{array}\right)\prod_{i=1}^{r}\left(k_{i}-1\right)!p^{k_{i}}. \end{array}$$

The Hessian matrix of second-order partial and cross-partial derivatives determines whether or not the likelihood equations indicated root is in fact a (local) maximum [21, 22]:

(12) $$\begin{array}{c} H\left(\hat{\theta }\right)=\left[\begin{array}{cccc} {\frac{\partial^{2}\ell }{\partial \theta_{1}^{2}}|}_{\theta =\hat{\theta }} & {\frac{\partial^{2}\ell }{\partial \theta_{1}\partial \theta_{2}}|}_{\theta =\hat{\theta }} & \cdots & {\frac{\partial^{2}\ell }{\partial \theta_{1}\partial \theta_{k}}|}_{\theta =\hat{\theta }}\\ {\frac{\partial^{2}\ell }{\partial \theta_{2}\partial \theta_{1}}|}_{\theta =\hat{\theta }} & {\frac{\partial^{2}\ell }{\partial \theta_{2}^{2}}|}_{\theta =\hat{\theta }} & \cdots & {\frac{\partial^{2}\ell }{\partial \theta_{2}\partial \theta_{k}}|}_{\theta =\hat{\theta }}\\ \vdots & \vdots & \ddots & \vdots \\ {\frac{\partial^{2}\ell }{\partial \theta_{k}\partial \theta_{1}}|}_{\theta =\hat{\theta }} & {\frac{\partial^{2}\ell }{\partial \theta_{k}\partial \theta_{2}}|}_{\theta =\hat{\theta }} & \cdots & {\frac{\partial^{2}\ell }{\partial \theta_{k}^{2}}|}_{\theta =\hat{\theta }} \end{array}\right]. \end{array}$$

In order to optimize the problem, we use bordered Hessian:

(13) $$\begin{array}{c} H\left(\Lambda \right)=\left[\begin{array}{cc} \frac{\partial^{2}\Lambda }{\partial \lambda^{2}} & \frac{\partial^{2}\Lambda }{\partial \lambda \;\partial x}\\ {\left(\frac{\partial^{2}\Lambda }{\partial \lambda \;\partial x}\right)}^{⊤} & \frac{\partial^{2}\Lambda }{\partial x^{2}} \end{array}\right]\\ =\left[\begin{array}{cc} 0 & \frac{\partial g}{\partial x}\\ {\left.\frac{\partial g}{\partial x}\right)}^{⊤}\frac{\partial^{2}\Lambda }{\partial x^{2}} \end{array}\right]. \end{array}$$

Table 2 presents the results of the classification process:

For each variable (response), a probability value is generated, revealing the degree to which it is interdependent with its class and hence the direction in which each question has an effect. In other words, a first classification of the responses into distinct categories can define the options and skills of each student. In this example, based on the questionnaire, three classes were used (theoretical direction, positive direction, and technological direction), where the students were classified based on their answers and the algorithm of the DAG used.

### 3.2. Step 2: Differential Privacy and Results

On the contrary, in order to protect an individual who is deciding to allow their data to be included in the repositories that proposed the method, we use differential privacy. Let *q* be a counting query. Trying to protect privacy by adding noise results in [3, 23–25],

(14) $$\begin{array}{c} M\left(x\right)=q\left(x\right)+\text{noise.} \end{array}$$

The Laplace distribution with scale parameter *b* > 0 (assuming position parameter 0) is defined as the distribution with probability density function:

(15) $$\begin{array}{c} \text{Lap}\left(x|b\right)=\frac{1}{2b}e^{-\left|x\right|/b}. \end{array}$$

So, it turns out

(16) $$\begin{array}{c} \mathrm{Pr}\left[M\left(x\right)\in S\right]=\mathrm{Pr}\left[M\left(x\right)\in S|\text{enoughnoise}\right]+\mathrm{Pr}\left[M\left(x\right)\in S|\text{notenoughnoise}\right]\leq e^{\varepsilon }\mathrm{Pr}\left[M\left(y\right)\in S\right]+\delta . \end{array}$$

The *l* 1-sensitivity of a function *f* is calculated as

(17) $$\begin{array}{c} \Delta =\underset{x∼x^{\prime }}{\max}f\left(x\right)-f\left(x^{\prime }\right). \end{array}$$

For example, compare the *x* database with the test scores and the query for the average score:

(18) $$\begin{array}{c} q\left(x\right)=\frac{\sum_{i=1}^{n}x_{i}}{n}. \end{array}$$

If we use a neighborhood type relationship such as |*x*_*i*_ − *x*_*i*_′| ≤ *x*_max_, then the sensitivity of the question will be

(19) $$\begin{array}{c} \Delta =\underset{x∼x^{\prime }}{\max}\left|q\left(x\right)-q\left(x^{\prime }\right)\right|\\ =\frac{1}{n}\underset{x_{i},x_{i}^{\prime }}{\max}\left|x_{i}-x_{i}^{\prime }\right|i\in \left[1,n\right]. \end{array}$$

According to the above equation, the differential privacy mechanism will be

(20) $$\begin{array}{c} M\left(x\right)=\frac{\sum_{i=1}^{n}x_{i}}{n}+\text{Lap}\left(\frac{x_{\max}}{n\in }\right). \end{array}$$

Finally,

(21) $$\begin{array}{c} Pr\left[\text{notenoughnoise}\right]\leq Pr\left[\text{Lap}\left(\mu ,b\right)\leq 2\right]+Pr\left[\text{Lap}\left(\mu ,b\right)\leq 1\right]=\\ =\frac{1}{2}\text{exp}\left(\frac{2-\mu }{b}\right)+\frac{1}{2}\text{exp}\left(\frac{1-\mu }{b}\right)\leq \text{exp}\left(\frac{2-\mu }{b}\right). \end{array}$$

To prove that the proposed differential privacy system is secure against level 2 attacks, we need to prove that it does not allow distance calculation. Specifically, assuming that a DRE E is used to encrypt the DB to get *E*(DB), a level 2 attacker with *H* = 〈E (DB), P, I〉 can retrieve DB if P contains at least *d* + 1 points *x*_i_ (1 ≤ *i* ≤ *d* + 1) so that the set of vectors {*x*_j_ − x_1_|2 ≤ *j* ≤ *d* + 1} is linearly independent. A hash function used by the Distributed Hash Table (DHT) to assign file ownership to network nodes which generates a key of 256 bits, which is enough to withstand the level 2 attack on the DRE. This system's encryption function hides the distance between two points in a database table; therefore, it must be determined which of the two points is closest to a query point *q*, and it must also be implemented [4, 26]:

(22) $$\begin{array}{c} d\left(p1,q\right)\geq d\left(p2,q\right)\sqrt{{\left\|p1\right\|}^{2}-2p1*q+{\left\|q\right\|}^{2}}\geq \sqrt{{\left\|p2\right\|}^{2}-2p2*q+{\left\|q\right\|}^{2}}{\left\|p1\right\|}^{2}-{\left\|p2\right\|}^{2}+2\left(p1-p2\right)*q\geq 0. \end{array}$$

where ||p|| represents the Euclidean norm of *p*, represents the gradient system, and ||p||2 can be represented by *pp*. As a result, the problem of inequality can be broken down into a slew of gradient calculations. This shows that Espe's product conservation is being assessed in terms of encryption, i.e., ∀p1, p2 ∈ DB, p1 *p*2 = Espe (p1, K) Espe (p2, K), to calculate k-NN [24, 27].

The attacker cannot increment the estimate of P to diminish the likelihood of a collision and rehash the attack as, within the proposed design, the item maintenance encryption is not remotely retrievable as [28, 29]

(23) $$\begin{array}{c} f\left(p1^{\prime },p2^{\prime }\right)=\sqrt{p1^{\prime }*p1^{\prime }-2\left(p1^{\prime }*p2^{\prime }\right)+p2^{\prime }*p2^{\prime }}\neq d\left(p1^{\prime },p2^{\prime }\right). \end{array}$$

To put it another way, if the encryption E (i.e., E is DRE), then a computing technique *f* such that, for all points in time, the differential privacy function ET (i.e., ET is DRE) cannot be remotely retrieved, *p*_1_ and *p*_2_ and any encryption key K_1_; it holds that *a*_1_ = E (*p*_1_, K_1_) and *a*_2_ = E (*p*_2_, K_1_); we have *f* (*a*_1_, *a*_2_) = *d* (*p*_1_, *p*_2_). That is, the distance *d* (p1, p2) may be determined from the encrypted values a1 and a2 regardless of the encryption key.

### 3.3. Step 3: Recommendation System

Finally, an intelligent recommendation memory-based approach was used to measure user privacy and compute the similarity between users. It is a neighborhood-based collaborative filtering approach to produce recommendations [11–13]:

(24) $$\begin{array}{c} r_{u,i}={\text{aggr}}_{u^{\prime }\in U}r_{u^{\prime },i}. \end{array}$$

The top *N* most comparable users to user *u* who share the same level of privacy as user *i* are denoted by *U*. The aggregation function includes

(25) $$\begin{array}{c} r_{u,i}=\frac{1}{N}\sum_{u^{\prime }\in U}r_{u^{\prime },i}r_{u,i}\\ =k\sum_{u^{\prime }\in U}\text{simil}\left(u,u^{\prime }\right)r_{u^{\prime },i}, \end{array}$$

where *r*_*u*_ is the average privacy of user *u* for all the users rated by *u*.

The suggested technique determines the cosine similarity between two users in a neighborhood-based approach [4, 6, 30]:

(26) $$\begin{array}{c} \text{simil}\left(x,y\right)=\cos\left(\overset{⟶}{x},\overset{⟶}{y}\right)\\ =\frac{\overset{⟶}{x}\cdot \overset{⟶}{y}}{\left\|\overset{⟶}{x}\right\|\times \left\|\overset{⟶}{y}\right\|}\\ =\frac{\sum_{i\in I_{xy}}r_{x,i}r_{y,i}}{\sqrt{\sum_{i\in I_{x}}r_{x,i}^{2}}\sqrt{\sum_{i\in I_{y}}r_{y,i}^{2}}}. \end{array}$$

Figure 2 shows the performance results of the proposed method.

As seen in the information supplied above, these findings demonstrate a solid solution to the challenging problem of grouping students to execute tailored educational programs. With the widespread usage of intelligent approaches such as those used in this study, small and heterogeneous student groups can form with members of each group sharing comparable characteristics of student ability, learning difficulties, and psychosocial and cognitive profile. By quickly managing the student potential in their class, as well as being aware of each group's unique characteristics such as their interests, unique experiences, learning rhythms, and learning styles, the teacher can easily manage the student potential of their class and offer high-quality education, taking into account the specific educational needs and capabilities of each group. In addition, the algorithm may be utilized in traditional classrooms and digital or e-learning programs, facilitating the teaching role, as it can compensate for challenges in multicriteria grouping and differentiation of students in a wide range of subject areas. Additionally, it can be utilized with many pupils and produce results in a short amount of time, assuming that the required data is available. Another presumption supporting this idea is that the amount of data that can be regarded as quantitative data or the number of evaluable criteria that come from a comprehensive evaluation of a student is limitless. Finally, each student's talents are automatically classified into various groups. They were applying an AI technique known as directed acyclic graph learning. Each learner's private information is protected using differential privacy in the model. Collaborative filtering's intelligent module provides customized real-time privacy advice.

## 4. Conclusions

This study presented an innovative recommendation system for privacy-preserving education technologies. It is a hybrid intelligent computing system that can create learning programs based on the unique needs of each learner. It is based on advanced machine learning techniques for performing high-level privacy-preserving analyses to create learning repositories adapted to the trainees' skills and experiences. The instructional material of educational systems may be successfully rearranged depending on assessment criteria using this novel and privacy-preserving approach. Specifically, using machine learning and differential privacy, this study provides a directed acyclic graph approach to automatically classify each student into a category based on their skills. Next, the model takes advantage of differential privacy. This technology makes it possible to gather relevant information from databases containing the personal information of individuals without disclosing sensitive identification about each individual. Personalized real-time data are also provided by an intelligent suggestion process based on collaborative filtering.

The proposed intelligent system achieved remarkable results in all cases of evaluation, always taking into account the modeling difficulties and uncertainty introduced by the subjective learning system. An important innovation is related to using privacy-preserving recommendations capable of solving multidimensional and complex problems. Also, an exciting finding is emerged from this research related to the possibility of applying to truly unstructured data, techniques, and methodologies and derived from fully theoretical computing, with fully exploitable and realistic results. Furthermore, the proposed method uses a neighborhood-based methodology to determine the cosine similarity between two users as a significantly innovative approach.

Humans are prone to errors or biases that might skew results while doing repetitive tasks such as reading and analyzing open-ended survey replies and other text data. A few simple steps are required for natural language processing (NLP)-powered tools to be taught to the language and criteria of the educational process. So, once they get the machines up and running, they perform far better than humans could ever hope to accomplish. To keep up with the changing marketplace or the language of their education, NLP can be used to investigate and extend the model, which will allow the automated system to take full advantage of modeling learning systems' wider dependencies with greater accuracy and efficiency. Also, text analysis on a large scale on a variety of papers, internal systems, emails, social media data, online reviews, and more will be made possible by NLP technology. Data can be processed in a matter of seconds or minutes, compared to the days or weeks it would take to analyze manually.

## Figures and Tables

**Figure 1:** The proposed architecture.

**Figure 2:** Proposed model loss and accuracy.

**Table 1:** Statistical analysis of the preliminary test.

Quest	Mean	S	S*δ*	*r*_*δ*_	*R* ^2^	Cronbach a
Q1	3.425	1.659	5.456	0.799	0.887	0.879
Q2	3.376	1.544	5.433	0.711	0.806	0.806
Q3	3.125	1.355	5.562	0.798	0.890	0.811
Q5	2.788	1.678	6.226	0.542	0.651	0.870
Q7	3.115	1.454	5.987	0.794	0.874	0.806
Q8	3.089	1.599	5.998	0.789	0.799	0.798
Q9	3.341	1.473	5.887	0.801	0.888	0.783
Q10	3.184	1.932	5.752	0.732	0.801	0.797

**Table 2:** Classification results.

	OvAc (%)	AvAc (%)	Kappa	McNemar	*R* ^2^	RRSE
Class_1	99.44	98.67	0.8992	30.172	0.989	0.0459
Class_2	98.37	97.52	0.8885	29.674	0.981	0.0518
Class_3	99.12	98.33	0.8973	30.029	0.987	0.0479

## Data Availability

The data used to support the findings of the study are available from the corresponding author upon reasonable request.

## References

[1] Al-Dojayli M., Czekanski A. (2017). Integrated engineering design education: vertical and lateral learning. *Journal of Integrated Design and Process Science*.

[2] Alzubaidi L., Zhang J., Humaidi A. J. (2021). Review of deep learning: concepts, CNN architectures, challenges, applications, future directions. *Journal of Big Data*.

[3] D’Acquisto G., Domingo-Ferrer J., Kikiras P., Torra V., de Montjoye Y.-A., Bourka A. (2015). Privacy by design in big data: an overview of privacy enhancing technologies in the era of big data analytics. *ArXiv151206000 Cs*.

[4] Shen Z., Zhong T. (2021). Analysis of application examples of differential privacy in deep learning. *Computational Intelligence and Neuroscience*.

[5] del Águila I. M., del Sagrado J. (2016). Bayesian networks for enhancement of requirements engineering: a literature review. *Requirements Engineering*.

[6] Mrad A. B., Delcroix V., Piechowiak S., Leicester P., Abid M. (2015). An explication of uncertain evidence in Bayesian networks: likelihood evidence and probabilistic evidence. *Applied Intelligence*.

[7] Canbek G., Sagiroglu S., Temizel T. T., Baykal N. Binary classification performance measures/metrics: a comprehensive visualized roadmap to gain new insights.

[8] Koyejo O. O., Natarajan N., Ravikumar P. K., Dhillon I. S. (2014). Consistent binary classification with generalized performance metrics. https://dblp.org/rec/conf/nips/KoyejoNRD14.html.

[9] Elmrabit N., Zhou F., Li F., Zhou H. Evaluation of machine learning algorithms for anomaly detection.

[10] Bringer J., Chabanne H., Patey A. (2013). Privacy-preserving biometric identification using secure multiparty computation: an overview and recent trends. *IEEE Signal Processing Magazine*.

[11] Aggarwal C. C., Aggarwal C. C. (2016). Neighborhood-based collaborative filtering. *Recommender Systems: The Textbook*.

[12] Deschênes M. (2020). Recommender systems to support learners’ Agency in a Learning Context: a systematic review. *International Journal of Educational Technology in Higher Education*.

[13] Isinkaye F. O., Folajimi Y. O., Ojokoh B. A. (2015). Recommendation systems: Principles, methods and evaluation. *Egyptian Informatics Journal*.

[14] Alallawi B., Denne L., Apanasionok M. M., Grindle C. F., Hastings R. P. (2021). Special educators’ experiences of a numeracy intervention for autistic students. *European Journal of Special Needs Education*.

[15] Demetriou A., Spanoudis G., Mouyi A. (2011). Educating the developing mind: towards an overarching paradigm. *Educational Psychology Review*.

[16] Klašnja-Milićević A., Ivanović M. (2021). E-learning personalization systems and sustainable education. *Sustainability*.

[17] Cha H. J., Ahn M. L. (2014). Development of design guidelines for tools to promote differentiated instruction in classroom teaching. *Asia Pacific Education Review*.

[18] Korkmaz C., Correia A.-P. (2019). A review of research on machine learning in educational technology. *Educational Media International*.

[19] Abbitt J. T., Boone W. J. (2021). Gaining insight from survey data: an analysis of the community of inquiry survey using Rasch measurement techniques. *Journal of Computing in Higher Education*.

[20] Berger J. O., Berger J. O. (1985). Bayesian analysis. *Statistical Decision Theory and Bayesian Analysis*.

[21] Mahmud M. S., Huang J. Z., Salloum S., Emara T. Z., Sadatdiynov K. (2020). A survey of data partitioning and sampling methods to support big data analysis. *Big Data Mining and Analytics*.

[22] Blyumin S., Pogodaev A., Khabibullina E. Graph-structural modeling of some special organizational systems.

[23] Alshalali T., M’Bale K., Josyula D. Security and privacy of electronic health records sharing using hyperledger fabric.

[24] Hou R., Tang F., Liang S., Ling G. (2021). Multi-Party Verifiable Privacy-Preserving Federated k-Means Clustering in Outsourced Environment. *Security and Communication Networks*.

[25] Li Z., Xu W., Shi H., Zhang Y., Yan Y. (2021). Security and privacy risk assessment of energy big data in cloud environment. *Computational Intelligence and Neuroscience*.

[26] Behera S., Prathuri J. R. Application of homomorphic encryption in machine learning.

[27] Su X., Khoshgoftaar T. M., Greiner R. Imputed neighborhood based collaborative filtering.

[28] Bordel B., Alcarria R., Robles T. (2022). Lightweight encryption for short-range wireless biometric authentication systems in Industry 4.0. *Integrated Computer-Aided Engineering*.

[29] Iezzi M. Practical privacy-preserving data science with homomorphic encryption: an overview.

[30] Fu Q., Tian Y., Sun J. (2021). Modeling and simulation of dynamic lane reversal using a cell transmission model. *Journal of Intelligent Transportation Systems*.

